# Analysis of Dietary Supplement Use and Influencing Factors in the Mongolian Population

**DOI:** 10.1155/2022/4064588

**Published:** 2022-03-22

**Authors:** Zhidi Wang, Wuyun Tana Li, Yumin Gao, Xin Xue, Hui Pang, Wenli Hao, Yuan Xia, Shiqi Wang, Xiong Su, Lingyan Zhao, Minhui Li

**Affiliations:** ^1^Inner Mongolia Medical University, Hohhot, China; ^2^Laboratory for Molecular Epidemiology in Chronic Diseases, Inner Mongolia Medical University, Hohhot, China; ^3^Inner Mongolia Autonomous Region Hospital of Traditional Chinese Medicine (Clinical College of Traditional Chinese Medicine of Inner Mongolia Medical University), Hohhot, China; ^4^Inner Mongolia Autonomous Region Institute of Chinese and Mongolian Medicine, Hohhot, China

## Abstract

**Objective:**

Dietary supplements (DS) may improve micronutrient deficiencies, but the unique eating habits and cultural customs of the Chinese Mongolian population affect their choice of DS. Therefore, this study adopted a cross-sectional method to explore the current status of DS use and to assess the influencing factors in the Mongolian population in Inner Mongolia, China.

**Methods:**

We used a multistage random cluster sampling method to select 1,434 Mongolian people aged ≥ 18 years in Hohhot and Xilinhot, Inner Mongolia. Data regarding general patient characteristics and DS use through questionnaire surveys were obtained, and the blood plasma was collected for biochemical index detection. The binary logistic regression and decision tree algorithm were used to predict the factors influencing DS use among the Mongolian population.

**Results:**

Among 1,434 participants that completed the baseline survey, the usage rate of DS was 18.83%, and more women than men used DS (*P* = 0.017). Higher use of DS was reported among individuals aged ≤ 34 years, but this difference is not statistically significant (*P* = 0.052). Usage rate was higher among those living in urban areas (*P* < 0.001), those with higher education (*P* < 0.001), those engaged in mental work (*P* < 0.001), and nonsmokers (*P* = 0.019). The biochemical test results showed that the proportion of people with abnormal total cholesterol levels using DS was lower (*P* = 0.003), but that of those with abnormal triglyceride levels using DS was higher (*P* = 0.001), compared with the proportion of those with normal levels in each case. The most commonly used supplement was calcium (58.15%). Education level was the main factor affecting DS intake. The results of the binary logistic regression model and decision tree model both showed that region, educational level, and abnormal triglyceride levels were significant factors influencing DS intake among Mongolians.

**Conclusion:**

Findings from this study indicate that DS intake is uncommon in the Mongolian population. In addition, sex, region, education level, and triglyceride levels may influence DS use.

## 1. Introduction

Currently, there is no global consensus on the definition of dietary supplements (DS) [1]. The United States Food and Drug Administration, under the Dietary Supplement Health and Education Act promulgated in 1994, defines DS as products intended to supplement the diet, including vitamins, minerals, herbs, amino acids, enzymes, and other ingredients, which are intended to be used in form of pills, capsules, tablets, or liquids [2]. However, there is no clear legal definition of the term in China. As the economy and living standards have improved, people are paying more attention to their health; however, it is difficult for laypeople to decide whether they need DS and how to choose them.

Globally, the sales of DS reached $128 billion in 2007 [3], although the prevalence of use varies greatly among different countries. The use of DS may be affected by factors such as demographics, cultural customs, lifestyle, and eating habits. Previous studies have shown that women, older people, and people with higher education are more likely to use DS [4–7]. In addition, it has been reported that people using DS have healthier eating habits, are nonsmokers [8], are physically active [5], and tend to eat more fruits and vegetables [9]. In contrast, people who do not use DS prefer high-fat, low-fiber diets [9]. According to previous survey data, the prevalence of DS use in the United States is 52% [10], while the prevalence in the Polish population is 77.84% [11]; however, in some Asian countries, such as South Korea and Japan, the prevalence of DS use in adults is low [12, 13]. In China, there are limited research data on the use of DS among Mongolian people in Inner Mongolia. A cross-sectional study on nutrition and health monitoring reported that the usage rate of DS in the population aged 6 years and over in China was only 0.71% [14].

China has a diverse population comprising 56 ethnic groups. Among them, the Mongolian people are considered ethnic minorities, accounting for 8% of the total Chinese population. Unlike the Han ethnicity, Mongolians have a unique diet and lifestyle. For example, they tend to consume more animal fat and alcohol, while consuming less grains, fresh vegetables, and beans [15]. Studies have shown that unbalanced eating habits decrease the level of vitamins and minerals, which are insufficient for maintaining the body's normal functions, and eventually cause scurvy, beriberi, pellagra, rickets, osteoporosis, and other vitamin deficiencies [16, 17]. In a survey of adult residents in the United States, about 23% of DS consumers were advised by health care professionals to improve their physical condition and maintain their health [18].

Commonly used DS include fish oil, omega-3 fatty acids, and multivitamins and minerals (such as calcium, iron, and selenium) [19]. People often use DS to reduce weight, supplement energy, and improve the state of undernutrition or deficiency caused by drugs or a poor diet [20, 21]. In addition, they can potentially reduce the incidence and related risks of some chronic conditions and diseases such as cognitive impairment, cardiovascular disease, and cancer [22]. DS also play an important role during certain periods. For example, some pregnant women use vitamins during pregnancy to prevent adverse maternal and child outcomes, including spontaneous abortion, preeclampsia, low birth weight, and developmental abnormalities [23, 24]. In infancy, the American Academy of Pediatrics recommends that breastfed infants older than 4 months receive iron supplementation before introducing iron-containing complementary foods and that all exclusively breastfed infants receive vitamin D supplementation [25]. However, improper selection and consumption of DS may have adverse effects on the body. For example, excessive calcium intake can lead to an increase in the incidence of cardiovascular diseases, excessive consumption of vitamin E may cause diarrhea, weakness, blurred vision, and gonadal dysfunction, and excessive amounts of vitamin A are associated with decreased bone density and increased fracture risk. In addition, some side effects of anabolic steroids include cardiomyopathy, changes in blood lipids, acne, and liver toxicity [1, 2, 26, 27].

Currently, there is no research on the use of DS in the Mongolian population in China, and the views of the Chinese ethnic minority populations on DS use remain unclear. Therefore, this study is aimed at assessing the prevalence of DS use in the Mongolian population and at determining their specific demographic and lifestyle characteristics. This will enable us to fill in some gaps regarding DS use among ethnic minorities in China and provide the targeted scientific basis for the formulation of DS-related guidelines and policies for Mongolian minority areas.

## 2. Materials and Methods

### 2.1. Study Sample

This was an observational, cross-sectional study that used multistage stratified cluster sampling. The study was conducted in Hohhot and Xilinhot cities, which are located in the Inner Mongolia Autonomous Region. Five communities were selected from the two cities. A total of 1,434 Mongolian adults (537 men and 897 women) volunteered to participate in this investigation from July 2019 to August 2020. The study was approved by the Ethics Review Committee of Inner Mongolia Medical University, and all participants signed an informed consent form before the investigation. The epidemiological investigation process is presented in Figure 1.

#### 2.1.1. Inclusion Criteria

Inclusion criteria are as follows:

- Mongolian ethnicity
- Aged ≥ 18 years
- Able to complete the questionnaire correctly (defined as being able to understand Mongolian or Chinese and be able to make judgments about problems, and without comprehension, expression, and hearing impairments.)

#### 2.1.2. Exclusion Criteria

Exclusion criteria are as follows:

- Patients with mental illness
- Pregnancy or lactation
- Patients with language impairment caused by serious diseases

### 2.2. Variables

All investigators were uniformly trained to use the self-designed questionnaires for face-to-face interviews in Chinese or Mongolian language and to use the measurement instruments. A 20-item questionnaire was developed to evaluate the prevalence of DS use and the characteristics of the users. The questionnaire was pretested in a pilot study and was distributed to 200 research participants. After the pilot survey, analyses of the reliability and validity of the pretest survey results were carried out. The SPSS test results showed that Cronbach's coefficient *α* was 0.744 (>0.700), indicating that the questionnaire had good reliability, and the Kaiser–Meyer–Olkin value was 0.657 (>0.600), indicating that the validity of the questionnaire was acceptable.

At the beginning of the questionnaire, the participants were asked to state their ethnicity. Those who belonged to the Mongolian ethnicity were the focus of this research and were asked to proceed to the first section of the questionnaire. The survey comprised three sections: (1) demographic factors: this section of the questionnaire included demographic information such as the participants' age, sex, level of education, occupation, smoking status, alcohol use, sleep quality, dietary habits (vegetarian or nonvegetarian), anthropometric measurements, and self-reported health conditions (including diabetes mellitus, hypertension, coronary heart disease, and stroke); (2) DS consumed: the participants were asked, “Have you used any type of DS in the past 1 year?” If the participant responded “Yes,” the information regarding the DS type was recorded; and (3) biochemical indexes: venous blood (5 mL) was drawn from each participant into an ethylenediamine tetraacetic acid (EDTA) anticoagulant tube in the morning after 8 hours of fasting, the plasma was collected after centrifugation, and fasting blood glucose and blood lipids (including uric acid, triglycerides (TG), total cholesterol, high-density lipoprotein (HDL), and low-density lipoprotein (LDL)) were measured.

### 2.3. Assessment of Covariates

Anthropometric measurements include the assessment of height, weight, waist circumference, and hip circumference. When measuring the height and weight, the participants were required to wear coats, not wear a crown and shoes, stand with their heels closed at 45 degrees between the feet, and stand with heels close to the height rod. The height data record was accurate to 0.1 cm, and the weight data record was accurate to 0.1 kg. Body mass index (BMI) was calculated as weight (kg) divided by height (m^2^) (based on the Group of China Obesity Task Force definition of BMI stratification standards: <18.5 for underweight, 18.5–23.9 for normal weight, 24.0–27.9 for overweight, and ≥28.0 for obese).

Waist and hip measurements required participants to stand with their feet 25–30 cm apart and remove their outer clothes. Then we measured the waist circumference by putting a measuring tape around the waistline at 0.5–1 cm above the umbilicus. For obese people, measurement was taken at the thickest part of the waist. The hip reading is the measurement of the horizontal circumference of the body at the most prominent point of the buttocks. Both data records were accurate to 0.1 cm.

### 2.4. Statistical Analyses

The EpiData 3.1 software was used for data entry, and statistical analyses were performed using SPSS 25.0 (IBM, New York, USA). Categorical variables were compared using the *χ*^2^ test. The usage rates of different types of DS are expressed as percentages (%). The demographic variables were analyzed using bivariate logistic regression (enter method) to determine which of these univariates were significantly associated with DS use. In addition, we calculated the odds ratio (OR; OR = 1: there is no relationship between the factor and the dependent variable; OR > 1: the variable is a risk factor; and OR < 1: the variable is a protective factor) and 95% confidence interval (CI). Categorical variables were used in this study; therefore, the chi-squared automatic interaction detection (CHAID) decision tree algorithm was used to predict the main factors influencing DS use in the Mongolian population. The MedCalc V19.6.3 software was used to create and compare the receiver operating characteristic (ROC) curve of the logistic regression model and the decision tree model. All statistical tests were two-sided, and the significance level was set at 0.05.

## 3. Results

In total, 1,434 Mongolian individuals who met the inclusion criteria were enrolled in this study. The average age of the participants was 52.61 ± 14.38 (range 18–83) years. Among them, the 55–64-year age group had the largest proportion of the participants, and women accounted for 62.55% of the study sample. In this study, most Mongolians were from rural areas (51.81%), while the rest were from urban (25.03%) and pastoral areas (23.15%). The highest education level was mainly junior or senior high school (47.28%), followed by the primary school or lower (39.21%). Of the 1,434 participants, 50.14% were engaged in occupations involving physical effort and 17.57% in occupations involving mental effort, while the remaining participants were unemployed or retired.

### 3.1. General Information about the Research Participants

Table 1 shows the sociodemographics, lifestyle, and disease history of DS users and nonusers. Approximately 18.83% of the participants reported using DS for more than 3 months in the previous year. In total, 15.64% of men and 20.74% of women used DS (*P* = 0.017). A higher proportion of people living in urban areas (23.40%) reported using DS, while people in pastoral areas used less DS (8.43%) (*χ*^2^ = 31.264, *P* < 0.001). The results also showed that the higher the education level, the higher the frequency of DS use (*χ*^2^ = 33.880, *P* < 0.001). Additionally, those with occupations requiring mental effort (26.98%) and people who were unemployed or retired (21.81%) had a higher DS usage rate than those engaged in occupations requiring physical effort (*χ*^2^ = 24.422, *P* < 0.001). Regarding lifestyle choices, the highest percentage of DS users were from the nonsmoker group (20.75%). There were no significant differences in the DS usage in terms of age, vegetarian status, BMI, abdominal obesity, alcohol use, sleep quality, or history of diseases.

Table 2 shows the use of DS based on biochemical testing indicators. In our study, people with normal total cholesterol levels had a higher DS usage rate (20.39%) than those with abnormal levels (12.96%) (*χ*^2^ = 8.594, *P* = 0.003). However, the rate of DS usage was higher in people with abnormal TG levels than in those with normal TG levels, and the difference was significant (*χ*^2^ = 10.084, *P* = 0.001).

### 3.2. Logistic Regression to Analyze the Influencing Factors for DS Use

Logistic regression was used to evaluate the impact of demographic characteristics, lifestyle choices, and abnormal biochemical indicators on the likelihood of DS use (Table 3). The results showed that region, education level, and TG level were the significant factors influencing DS use. Compared with Mongolian people living in urban areas, those living in rural and pastoral areas demonstrated less usage of DS (adjusted odds ratio (AOR) = 0.528, 95% confidence interval (CI): 0.313–0.889; AOR = 0.504, 95% CI: 0.317–0.802, respectively). People with a junior or senior high school education level and those with a college or higher education level were 3.112 times and 2.185 times, respectively, more likely to use DS than those with a primary school or lower education level (*P* = 0.005). Compared with people with normal TG levels, people with abnormal TG levels were more likely to use DS (*P* < 0.001). Furthermore, we found that people aged > 45 years were more likely to use DS than people aged ≤ 34 years, but this finding was not significant (*P* = 0.257).

### 3.3. CHAID Decision Tree Algorithm to Analyze Influencing Factors for DS Use

Eleven variables—sex, age, region, occupation, education, tobacco use, and abnormalities in total cholesterol, TG, HDL-cholesterol, LDL-cholesterol, and uric acid levels—were used as input variables, and the use of DS was designated as a predictor in the building of the decision tree prediction model. The partition settings were as follows: 80% for the training set and 20% for the test set. The maximum tree depth was 3, and the termination parameter was a minimum number of records in the parent and child branches of 100 and 50, respectively. The significance level of segmentation and merging was set at 0.05, and *P* values were adjusted using the Bonferroni method. The visual result of the decision tree included 3 layers, a total of 12 nodes, and 7 paths. A total of 4 explanatory variables were screened out, namely education level, TG abnormalities, region, and sex. The results revealed that the education level was the most important factor influencing DS use among the Mongolian population; the path classification rules are presented in Figure 2.

### 3.4. Comparison of Two Forecasting Models

Separate ROC curves were created for the two models. For the logistic regression model, the results revealed an area under the curve (AUC) of 0.695 (95% CI: 0.670–0.719) and a standard error of 0.0171, while for the decision tree model, the AUC was 0.675 (95% CI: 0.650–0.699), and the standard error was 0.0175. The *Z*-test was used for comparison, and the results revealed that the difference in the predicted value of the two models was not significant (*Z* = 1.604, *P* = 0.108). These findings are shown in Figure 3.

### 3.5. Distribution of DS Types among Mongolians

Figure 4 shows that the most commonly used supplements were calcium (58.15%), vitamin C (8.52%), and multivitamins (8.15%). People who consumed other types of DS accounted for 13.70%, including those who consumed fish oil, Chinese herbal medicine, and other supplements. The supplements used in less than 5% of the participants included vitamin B, multivitamin/minerals, protein, vitamin E, and vitamin D.

## 4. Discussion

This study found that 18.83% of Mongolians use DS in China's Inner Mongolia region and the types of DS used in descending order of prevalence were calcium, vitamin C, multivitamins, vitamin B, multivitamins/minerals, protein, vitamin E, and vitamin D. Region, education level, and TG level were the main factors affecting the use of DS.

In recent years, the global consumption of DS has shown an upward trend. According to most consumers, the purpose of buying DS is to “improve” and “maintain” overall health [28–31], and DS use is receiving increasing attention. Vitamins and minerals are generally expected to promote good health and reduce the risk of chronic diseases, but the therapeutic efficacy of DS remains controversial. The results of a previous randomized double-blinded controlled trial revealed that supplementation with adequate multivitamins and minerals can reduce the blood pressure and serum C-reactive protein levels in obese women with an increased risk of cardiovascular disease [32]. However, other studies have shown that DS have no obvious effect on the treatment of hypertension, coronary heart disease, or cancer [33–35].

Calcium supplementation was very popular among the Mongolian population in our study. Calcium is an important component of the human body. Dietary calcium is mainly absorbed in the small intestine and finally deposited in the bones [36]. The functions of calcium involve strengthening the bones and teeth, regulating neuromuscular excitability, releasing various hormones and neurotransmitters, and playing a role in the process of blood coagulation [37–39]. In previous studies, it was found that a decrease in calcium level is not the only reason why people buy calcium supplements; age, sex, race, income, and other health problems (such as lower BMI, smoking cessation, and drinking) influence calcium supplement intake [40, 41]. Adequate calcium intake is important for the formation and maintenance of bone density [42]. Moreover, calcium supplementation can prevent many diseases, such as osteoporosis, cardiovascular disease, gastrointestinal disease, and kidney stones [26]. Owing to advertising and other marketing methods, the public generally believes that calcium is always good for health [43]. Therefore, calcium supplements have dominated the market in recent years, and millions of men, women, and children who wish to improve their bone health use calcium supplements. The results of this survey showed that the highest rate of calcium supplementation among Mongolians using DS was 58.15%, which is similar to the results of other studies on the use of DS in China, with calcium being the most popular DS [44, 45].

The utilization rate of vitamin C among the Mongolian population in this study was second to that of calcium. Vitamin C is an important antioxidant with anti-inflammatory and immune-enhancing effects [46]. The results of preclinical and observational studies in trauma, ischemia/reperfusion, and sepsis models have revealed that vitamin C administered in therapeutic doses can reduce oxidative stress and inflammation and restore endothelial and organ functions [47, 48]. The extensive use of vitamin C may be related to the dietary structure of the Mongolian population. The Mongolian diet is mostly based on meat. The proportion of fruits and vegetables is small, and the dietary vitamin C intake is low [49]; therefore, dietary vitamin C deficiency is rectified by supplementation. The usage rate of multivitamins was similar to that of vitamin C. Though vitamins are needed by the human body, the long-term health benefits of multivitamins are uncertain [50, 51]. The results of this study showed that a small proportion of the Mongolian population who used DS chose multivitamin supplements to maintain their health.

Our results revealed that the Mongolian DS usage rate was 18.83%, which is higher than the rate (0.71%) reported by Gong et al. in a large cross-sectional study among a Chinese population [14]. However, further studies are required to know whether it can meet the nutritional needs of the Mongolian population. Previous studies have shown that some Chinese people are at risk of insufficient intake of vitamin A, vitamin B, vitamin E, iron, phosphorus, and zinc [52]; in this study, the usage rates of vitamin B, vitamin D, vitamin E, protein, and multivitamin/minerals were all less than 5%. Therefore, more attention should be paid to micronutrient deficiencies among the Mongolian population in China. For those who are unable to obtain sufficient nutrients from food, the use of DS is a proven and reliable way of ensuring adequate nutrient intake to maintain and improve health [53].

This study included data on sex, age, region, education level, occupational status, smoking, drinking, biochemical indicators, and other indicators of the Mongolian participants and analyzed their relationship with the use of DS. The results showed that age had no significant influence on the use of DS. This finding differs from that of previous studies, which revealed that older adults are more likely to use DS than their younger counterparts [10, 52]. This may be because the age ranges of the research participants were different—our research participants were aged ≥ 18 years. We found that some demographic characteristics were related to the use of DS in the Mongolian population. The decision tree and logistic regression models revealed region and education to be the factors that influenced DS use among the Mongolian population in this study, with education level being the main influencing factor. Those with an education level of junior high school and above and urban residents were more inclined to use DS. People with higher education may have greater health awareness. Compared with residents of pastoral areas, urban and rural residents may have higher incomes and purchasing power as well as more accessibility to obtain DS. Some studies have proved that the education level and living area affect buying behavior [8, 14, 40, 54]. This suggests that clinicians need to strengthen health education among the Mongolian people with low education and those living in rural and pastoral areas to enhance their awareness of health care and the rational use of DS. Our results show that the use of DS is related to TG levels. Studies have shown that the intake of fish oil, omega-3 fatty acids, vitamin D, and other supplements can effectively reduce TG levels [55, 56]. Therefore, Mongolians with abnormal TG levels may potentially use DS instead of prescription drugs to reduce blood lipid concentrations. Furthermore, the decision tree model screened out sex, another influencing factor, from the logistic regression model. This is consistent with the results from previous studies, where women have been found to be more likely to use DS compared to men [28, 52]. The difference between the two models is that the decision tree model exposes interactions between variables, while the logistic regression model stratification reduces the sample size at each level. Furthermore, the test methods used by the two models differ [57]. The AUC of the ROC curve is used to compare the prediction effects of the two models. The AUC of the logistic regression model was slightly larger than that of the decision tree model, although the difference was not significant. Studies have shown that logistic regression and decision tree models complement each other and that the combination can more comprehensively explain the relationship between research variables [58].

There are some limitations to this study. First, we did not investigate the reasons for the intake of DS among the Mongolian people. Second, we did not accurately calculate the intake of various nutrients and, consequently, could not determine whether the overall nutritional intake of Mongolians was appropriate. Finally, even though the reliability and validity of our questionnaire are acceptable, the results were self-reported by the research participants, which may lead to recall bias and inaccurate results. However, the results of this study can provide an overview of, and the main influencing factors for, the use of DS among the Mongolian population of Inner Mongolia in China; this should help improve this population's awareness and purchasing behavior pertaining to DS. More importantly, it provides a reference for nutrient monitoring and guidance for the ethnic minority groups in China.

## 5. Conclusion

In this study, we found that 18.83% of Mongolians used DS and that the use of DS was related to sex, region, education level, and TG level. Calcium was found to be a common supplement. Health professionals should combine the existing knowledge and data on this topic to develop relevant manuals; in addition, health education aimed at the Mongolian people should be improved to establish an accurate understanding of DS. When sufficient nutrients cannot be obtained from the diet, effective guidance should be provided on the appropriate use of DS to promote health. Future research endeavors should encourage more regions and ethnic groups to explore the complexity of using DS, determine the appropriate way of using DS, and prevent abuse.

## Figures and Tables

**Figure 1:** Epidemiological investigation process of the cross-sectional study.

**Figure 2:** The results of the decision tree of the Mongolian dietary supplement use prediction model.

**Figure 3:** Comparison of ROC curves between the logistic regression model and decision tree model.

**Figure 4:** Frequency of Mongolian people using different types of dietary supplements.

**Table 1:** DS users and DS nonusers among Mongolian people by sociodemographic and lifestyle characteristics (*N* = 1,434).

Variables	DS users^a^	DS nonusers	*χ* ^2^	*P* value
	*N* (%)	*N* (%)		
Total	270 (18.83)	1164 (81.17)		
Sex (men)	84 (15.64)	453 (84.36)	5.702	0.017^∗^
Age				
≤34	45 (26.79)	123 (73.21)	9.404	0.052
35-44	38 (18.18)	171 (81.82)		
45-54	51 (15.60)	276 (84.40)		
55-64	82 (19.07)	348 (80.93)		
65^+^	54 (18.00)	246 (82.00)		
Region				
Urban	84 (23.40)	275 (76.60)	31.264	<0.001^∗^
Rural	158 (21.27)	585 (78.73)		
Pastoral areas	28 (8.43)	304 (91.57)		
Education^#^				
Primary school or lower	75 (13.54)	479 (86.46)	33.880	<0.001^∗^
Junior or senior high school	134 (19.48)	554 (80.52)		
College or higher	57 (33.33)	114 (66.67)		
Occupation				
Mental effort	68 (26.98)	184 (73.02)	24.422	<0.001^∗^
Physical effort	101 (14.05)	618 (85.95)		
Other	101 (21.81)	362 (78.19)		
BMI				
Underweight	8 (23.53)	26 (76.47)	5.922	0.115
Normal weight	98 (20.37)	383 (79.63)		
Overweight	101 (20.24)	398 (79.76)		
Obese	63 (15.00)	357 (85.00)		
Abdominal obesity	100 (17.45)	473 (82.55)	1.183	0.277
Vegetarian	8 (18.60)	35 (81.40)	0.001	0.970
Sleep problems	168 (19.00)	716 (81.00)	0.047	0.829
Diabetes	30 (19.87)	121 (80.13)	0.119	0.730
Hypertension	125 (17.43)	592 (82.57)	1.825	0.177
Coronary disease	16 (15.24)	89 (84.76)	0.956	0.328
Stroke	12 (16.44)	61 (83.56)	0.287	0.592
Tobacco use				
Daily smoker	34 (12.45)	239 (87.55)	9.932	0.019^∗^
Occasional smoker	4 (14.81)	23 (85.19)		
Ex-smoker	28 (18.54)	123 (81.46)		
Nonsmoker	204 (20.75)	779 (79.25)		
Alcohol use				
Daily drinker	11 (15.94)	58 (84.06)	0.742	0.690
Occasional drinker	68 (20.06)	271 (79.94)		
Non-drinker	191 (18.62)	835 (81.38)		

^∗^ *P* < 0.05. ^a^Use dietary supplements for three consecutive months in the past year. ^#^Missing data excluded.

**Table 2:** DS users and DS nonusers among Mongolian people by biochemical indicators' distribution (*N* = 1,434).

Variables	DS users^a^	DS nonusers	*χ* ^2^	*P* value
Total (%)	270 (18.83)	1164 (81.17)		
Total cholesterol abnormalities (%)	39 (12.96)	262 (87.04)	8.594	0.003^∗^
Triglycerides abnormalities (%)	166 (21.93)	591 (78.07)	10.084	0.001^∗^
HDL-cholesterol abnormalities (%)	128 (19.10)	542 (80.90)	0.063	0.802
LDL-cholesterol abnormalities (%)	40 (17.09)	194 (82.91)	0.550	0.458
Uric acid abnormalities (%)	62 (15.74)	332 (84.26)	3.399	0.065

^∗^ *P* < 0.05. ^a^Use dietary supplements for three consecutive months in the past year.

**Table 3:** Logistic regression analysis of the factors in dietary supplement use among Mongolian people.

Variables	Crude OR (95% CI)	Adjusted OR^a^ (95% CI)	*P* value^b^
Sex (vs. men)	1.411^∗^ (1.063, 1.875)	1.318 (0.928, 1.871)	0.123
Age (vs. ≤34)			0.257
35-44	0.600^∗^ (0.382, 0.942)	0.875 (0.500, 1.530)	
45-54	0.988 (0.624, 1.563)	1.484 (0.836, 2.633)	
55-64	1.188 (0.781, 1.807)	1.312 (0.811, 2.124)	
65^+^	0.932 (0.637, 1.363)	1.041 (0.688, 1.576)	
Region (vs. urban)			0.013^∗^
Rural	0.302^∗^ (0.191, 0.477)	0.528^∗^ (0.313, 0.889)	
Pasturing areas	0.341^∗^ (0.223, 0.522)	0.504^∗^ (0.317, 0.802)	
Education (vs. primary school or lower)			0.005^∗^
Junior or senior high school	3.193^∗^ (2.140, 4.766)	3.112^∗^ (1.568, 6.177)	
College or higher	2.067^∗^ (1.428, 2.992)	2.185^∗^ (1.216, 3.925)	
Occupation (vs. mental effort)			0.208
Physical effort	0.755 (0.529, 1.077)	1.025 (0.606, 1.732)	
Other	1.707^∗^ (1.259, 2.316)	1.341 (0.960, 1.874)	
Tobacco use (vs. daily smoker)			0.149
Occasional smoker	1.841^∗^ (1.245, 2.721)	1.628^∗^ (1.021, 2.596)	
Ex-smoker	1.506 (0.515, 4.403)	1.205(0.392, 3.700)	
Nonsmoker	1.150 (0.742, 1.783)	0.912 (0.552, 1.508)	
Total cholesterol abnormalities (vs. no)			0.071
Yes	0.581^∗^ (0.403,0.838)	0.638 (0.391, 1.039)	
Triglycerides abnormalities (vs. no)			<0.001^∗^
Yes	1.548^∗^ (1.181, 2.029)	2.029^∗^ (1.491, 2.935)	
HDL-cholesterol abnormalities (vs. no)			0.339
Yes	1.034 (0.793, 1.349)	1.153 (0.861, 1.545)	
LDL-cholesterol abnormalities (vs. no)			0.560
Yes	0.870 (0.601, 1.258)	1.157 (0.708, 1.891)	
Uric acid abnormalities (vs. no)			0.081
Yes	0.747 (0.547, 1.019)	0.740 (0.528, 1.038)	

^∗^ *P* < 0.05. ^a^All covariates in the table were mutually adjusted. ^b^*P* value after correction.

## Data Availability

The raw data supporting the conclusions of this article will be made available by the authors, without undue reservation.
